RETRACTED

# Protective Effect of Xinmailong Injection on Rats With Myocardial Infarction

**DOI:** 10.3389/fphys.2020.595760

**Published:** 2021-01-13

**Authors:** Wei Zhang, Kailiang Li, Yu Ding, Jiefeng Ren, Haijun Wang, Quanjin Si

**Affiliations:** Geriatric Cardiology Department of the Second Medical Center and National Clinical Research Center for Geriatric Diseases, Chinese PLA General Hospital, Beijing, China

**Keywords:** myocardial infarction, Xinmailong injection, protective effect, myocardial injury marker, rat model

## Abstract

This study aimed to investigate the protective effect of Xinmailong injection on rats with myocardial infarction. Thirty-six rats were induced myocardial infarction by operation, and six underwent sham operation. The myocardial infarction rats were randomly divided into three groups, 12 in each, and administered intraperitoneal injection of Xinmailong 5 mg/(kg·d), sodium creatine phosphate 80 mg/(kg·d), or normal saline as control respectively for 14 days. When the treatments were completed, the hemodynamic parameters of the rats were observed, and blood samples were taken to examine blood routine, blood coagulation index, liver and kidney function, inflammatory index, myocardial marker, thrombo-elastography, and other indicators. The morphology of cardiomyocytes was observed through light microscopy, and the microstructure of the myocardial cells was observed under electron microscope. No significant difference was found in blood routine, liver and kidney function, and blood coagulation index between the Xinmailong and sodium creatine phosphate groups compared with the saline control group. However, the inflammatory index and levels of myocardial markers were significantly decreased, and cardiac function was significantly improved. In terms of the morphology of myocardial cells, the Xinmailong group was similar to the sodium creatine phosphate group, the myocardial cell membrane was protected, and myocardial cell damage was reduced. In conclusion, Xinmailong is safe and had anti-inflammatory, heart-improving, and myocardial-protective effects. Its effectiveness is not inferior to that of sodium creatine phosphate.

## Introduction

Acute myocardial infarction (AMI) refers to myocardial necrosis caused by acute and persistent ischemia and hypoxia in coronary arteries. It can be complicated with arrhythmia, shock, or heart failure (HF) and often life-threatening. In the context of high incidence of metabolic diseases in modern society, the risk factors of cardiovascular diseases are poorly controlled. The AMI morbidity continues to increase every year. It is one of the leading causes of death in patients with cardiovascular diseases (Fox, 2000; Reynolds et al., 2017; Liu et al., 2019; Han et al., 2020). When AMI is complicated with HF, the inflammatory reaction following myocardial ischemia is more serious. Therefore, improving heart function, especially through early correction of abnormal cardiac function, is particularly important to improve patients’ quality of life. Xinmailong injection is a national class II medicine approved by China’s State Food and Drug Administration (CFDA) in 2006. It dilates coronary arteries, increases coronary blood flow, and improves microcirculation (Tang, 2008). A series of clinical trials performed in HF patients confirmed the effectiveness of Xinmailong in improving cardiac function, such as enhancement of myocardial contraction and inhibition of ventricular remodeling (Lu et al., 2018). It was reported that Xinmailong could inhibit platelet function and has antithrombotic activity, could be a potential therapeutic candidate to prevent or treat platelet-related cardiovascular diseases (Wang et al., 2019). Clinical outcome revealed that Xinmailong injection has certain protective effects on cardiac dysfunction. However, not many studies have been conducted on its myocardial protection effect. In this study, Xinmailong and control injections were administered to rats with myocardial infarction induced by left anterior descending coronary artery ligation, and the effect of Xinmailong injection was explored.

RETRACTED

## Materials and Methods

### Experimental Animals

Sixty adult male Wistar rats of clean grade from the Experimental Animal Center of the General Hospital of PLA were used (average body weight: 438 ± 38.6 g).

### Experimental Drug

Xinmailong injection was purchased from Yunnan Tengchong Pharmaceutical Factory (batch number: National Medicine Zhunzi Z20060443).

### Establishment of Myocardial Infarction Model

A total of 60 rats were anesthetized by injecting 3% pentobarbital sodium intraperitoneally, sham operation were performed on six, and left anterior descending coronary artery ligation were performed on the remaining 54. Acute myocardial ischemia was confirmed by ST elevation in ECG.

### Method of Administration and Grouping

Thirty six rats with myocardial infarction were randomly divided into three groups: the saline control group, the sodium creatine phosphate group, and the Xinmailong group, with 12 rats in each group. The drugs were administered through intraperitoneal injection, 80 mg/(kg·d) for the sodium creatine phosphate group, 5 mg/(kg·d) for the Xinmailong group, and equivalent volume of saline solution for control group for 14 days.

### Hemodynamic Assessment and Blood Test

After the experiment, the rats were anesthetized with 3% sodium pentobarbital and immobilized on the operating table with their backs down. The skin of the neck was cut, and the right carotid artery was exposed for arterial catheterization. A catheter containing 0.1% heparin sodium was inserted into the right carotid artery and then into the left ventricle through the right common carotid artery. Whether the cannula entered the ventricle was determined according to the change in the pressure pattern shown on display. The catheter was connected to the BL-420S biosignal acquisition system. Data including heart rate (HR), Left Ventricular Systolic Pressure (LVSP), Left ventricular end-diastolic pressure (LVEDP), maximal left ventricular pressure rising rate (+dP/dtmax), and maximal left ventricular pressure rising rate (−dP/dtmax) were recorded.

RETRACTED

After measuring the hemodynamic index, the rats were sacrificed. The blood was taken from the aorta to examine blood routine, blood coagulation indexes, liver and kidney functions, inflammatory indexes, myocardial markers, and other tests.

### Myocardial Cell Morphology and Ultrastructure

The left ventricular ring incision in each group was fixed with a 10% neutral formaldehyde buffer. Hematoxylin and eosin (HE) staining, Masson staining, microscopic examination, and tissue imaging were conducted. The myocardial tissue in the left ventricular ischemic area of the heart was excised, washed with normal saline, cut into 1-mm^3^ size, fixed in 2.5% glutaraldehyde, and observed under a transmission electron microscope for ultrastructural changes in the mitochondria of myocardial tissue.

### Statistical Methods

Statistical analysis was performed using SPSS 19.0 statistical software. Values were expressed as mean ± SD, and an *F*-test was used for comparison between groups. Value of *p* < 0.05 was considered statistically significant.

## Results

### Xinmailong Caused No Obvious Adverse Effect

During the course of the study, three rats died in both saline control and sodium creatine phosphate groups, while two died in the Xinmailong group. Therefore, at the end of the study, a total of nine rats in control group, nine in sodium creatine phosphate group and 10 in Xinmailong group were examined. We found no significant difference in body weight between the groups, and no significant differences were observed in white blood cell (WBC) count, neutrophil (N) count, platelet (PLT) count, hemoglobin (HB) content, and red blood cell (RBC) count between the groups, as shown in Table 1. In addition, no significant difference in coagulation parameters including thrombin time (TT), plasma-activated partial prothrombin time (APTT), plasma prothrombin activity (AA), and plasma fibrinogen (Fib) were found between the groups, as shown in Table 2. In general, Xinmailong caused no obvious adverse effect on animals, suggesting that Xinmailong is basically safe.

RETRACTED

**Table 1:** Comparative analysis of blood routine indicators between groups (*x̄* ± *s*).

Group	Number	WBC (×10^9^/L)	RBC (×10^12^/L)	Hb (g/dl)	PLT (×10^12^/L)	N
Sham	6	2.84 ± 0.72	8.94 ± 0.79	150.67 ± 17.43	990.33 ± 315.98	0.22 ± 0.12
Control	9	3.80 ± 1.14	9.11 ± 0.56	152.89 ± 12.97	911.89 ± 167.37	0.13 ± 0.08
Sodium creatine phosphate	9	3.12 ± 1.12	9.59 ± 0.88	159.67 ± 9.75	794.89 ± 114.37	0.14 ± 0.08
Xinmailong	10	3.18 ± 1.12	9.01 ± 0.69	152.60 ± 1.22	950.20 ± 87.54	0.15 ± 0.07

No significant differences in the indicators were noted between the groups.

**Table 2:** Comparative analysis of various indicators of coagulation routine between groups (*x̄* ± *s*).

Group	Number	TT (s)	APTT (s)	AA (%)	Fib (g/L)
Sham	6	31.97 ± 7.12	21.87 ± 2.31	55.83 ± 3.87	3.05 ± 0.22
Control	9	37.59 ± 10.44	22.71 ± 3.58	53.04 ± 6.04	2.93 ± 0.36
Sodium creatine phosphate	9	36.83 ± 4.13	21.87 ± 1.74	51.56 ± 4.82	2.56 ± 0.59
Xinmailong	10	31.62 ± 6.74	20.82 ± 1.76	52.80 ± 4.34	2.79 ± 0.28

No significant differences in the indicators were noted between the groups.

### Xinmailong Protects Myocardial Function While Suppresses Inflammation

We next measured serum creatine kinase (CK), CK-MB, type B natriuretic peptide (BNP), lactate dehydrogenase (LDH), aspartate aminotransferase (AST), alanine aminotransferase (ALT), creatinine (CRE), and C-reactive protein (CRP) to evaluate the myocardial function, liver function, kidney function, and inflammation levels. As expected, compared with sham group, the myocardial indicators such as CK, CK-MB, and BNP levels were significantly higher in saline control group, indicating that the heart damage is significant at the time of examination. Importantly, these indications in sodium creatine phosphate and Xinmailong injection group were significantly lower compare to control group, and not significantly different with that in sham operation group and between each other, suggesting that both treatments have myocardial protective effect, and they are similarly effective. The AST level was significantly increased in the saline control group compared with the sham operation group, and it is significantly decreased in sodium creatine phosphate and Xinmailong groups compared to control group. There was no significant difference between the sodium creatine phosphate and Xinmailong groups. Notably, compared with sham operation group, serum CRP level, the very important systematic inflammation indicator, was significantly increased in control group. Importantly, compare with saline control group, CRP level was significantly suppressed in creatine phosphate group and Xinmailong group, which showed no difference between sham and creatine phosphate group and Xinmailong group. These results suggest that AMI causes systematic inflammation, which can be suppressed by both sodium creatine phosphate and Xinmailong. Other indications including LDH, ALT, and CRE were not significantly different between groups (Table 3).

RETRACTED

**Table 3:** Comparative analysis of serum levels of C-reactive protein (CRP), aspartate aminotransferase (AST), creatine kinase (CK), CK-MB, type B natriuretic peptide (BNP), creatinine (CRE), alanine aminotransferase (ALT), and lactate dehydrogenase (LDH) levels in each group (*x̄* ± *s*).

Test items	Sham	Control	Sodium creatine phosphate	Xinmailong
number	6	9	9	10
CK	1072.5 ± 98.0^#^	1594.8 ± 93.5^*^	1239.6 ± 400.1^#^	1331.2 ± 343.6^#^
CK-MB	701.9 ± 134.3^#^	1085.1 ± 69.7^*^	898.4 ± 177.2^#^	733.7 ± 303.6^#^
BNP	331.4 ± 37.5^#^	508.3 ± 57.2 ^*^	361.6 ± 54.2^#^	371 ± 35.8^#^
LDH	1471.5 ± 140.3	1462.6 ± 134.9	1246.3 ± 335.9	1623.1 ± 625.8
CRP	0.025 ± 0.01	0.074 ± 0.02^*^	0.044 ± 0.03^#^^,^^*^	0.046 ± 0.01^#^^,^^*^
AST	110.2 ± 5.3	134.1 ± 10.5^*^	116.1 ± 17.7	126.9 ± 16.9
ALT	49.1 ± 2.8	52.8 ± 10.5	47.1 ± 5.1	43.3 ± 7.2
CRE	26.3 ± 1.8	27.8 ± 4.9	26.3 ± 4.4	26.9 ± 4.9

* Compared with the sham operation group, *p* < 0.05.

# Compared with the control group, *p* < 0.05.

We also performed comparative analysis on the indexes of thrombus elasticity. We found that the kinetics (K) value was significantly decreased and the angle value was significantly increased in the control, sodium creatine phosphate, and Xinmailong groups compared with the sham operation group. No statistically significant difference in the reaction time (R) and maximum amplitude (MA) values was observed between the groups (Table 4). These data suggest that AMI lead to abnormality of thrombus elasticity, which cannot be corrected by neither sodium creatine phosphate nor Xinmailong treatment.

**Table 4:** Comparative analysis of thromboelastogram in each group after the experiment (*x̄* ± *s*).

Group	Number	*R*	MA	*K* value	Angle
Sham	6	6.67 ± 2.28	64.7 ± 10.29	3.9 ± 0.85	45.98 ± 7.16
Control	9	6.46 ± 1.33	64.2 ± 12.46	1.96 ± 0.41^*^	66.54 ± 3.83^*^
Sodium creatine phosphate	9	5.33 ± 1.61	63.11 ± 12.07	2.27 ± 0.58^*^	68.08 ± 7.03^*^
Xinmailong	10	5.34 ± 3.36	52.89 ± 12.55	2.38 ± 1.55^*^	62.36 ± 14.83^*^

* Compared with the sham operation group, *p* < 0.05.

In addition to the serum biochemical indications, we also examine the hemodynamics-related indexes to evaluate the cardiac function. We found no statistically significant difference in the HR between the groups. In the comparison of LVEDP, LVSP, dp/dtmax, and −dp/dtmin, we found that in all the AMI groups (Control, Sodium creatine phosphate, and Xinmailong groups), LVEDP level was significantly higher, and LVSP, dp/dtmax, and −dp/dtmin were significantly lower than Sham operation group, suggesting compromised myocardial function in these animals. However, compare to control group, LVEDP level was significantly lower, and LVSP, dp/dtmax, and −dp/dtmin were significantly higher in sodium creatine phosphate and Xinmailong groups, suggesting both treatments preserved heart function. More importantly, in Xinmailong group LVSP level was significantly higher than in sodium creatine phosphate (Table 5). These data suggest that Xinmailong, as well as sodium creatine phosphate preserves cardiac function, and the effect of Xinmailong is not inferior to, and even better than sodium creatine phosphate in some aspects.

RETRACTED

**Table 5:** Comparative analysis of hemodynamics-related indexes in each group after the experiment (*x̄* ± *s*).

Group	Number	HR (bpm)	LVEDP (mmHg)	LVSP (mmHg)	dp/dtmax (mmHg/s)	−dp/dtmax (mmHg/s)
Sham	6	380.33 ± 13.88	2.42 ± 1.75	191.5 ± 4.68	13013.5 ± 324.14	7653.17 ± 452.63
Control	9	393.77 ± 16.75	19.56 ± 3.28^*^	168.44 ± 8.92^*^	9788.56 ± 754.67^*^	6045.67 ± 361.57^*^
Sodium creatine phosphate	9	389.67 ± 14.02	12.7 ± 4.73^*^^,^^#^	177.67 ± 7.42^*^^,^^#^	11849.67 ± 764.18^*^^,^^#^	7113.44 ± 351.43^*^^,^^#^
Xinmailong	10	384.5 ± 15.71	11.72 ± 3.44^*^^,^^#^	184.59 ± 5.47^*^^,^^#^^,△^	12058.78 ± 966.9^*^^,^^#^	7056.8 ± 573.21^*^^,^^#^

* Compared with the sham operation group, *p* < 0.05.

# Compared with the control group, *p* < 0.05.

∆ Compared with sodium creatine phosphate group, *p* < 0.05.

### Xinmailong Protects Myocardial Tissue

At 14 days post MI, Masson’s trichrome was performed to evaluate the overall cardiac injury, and the representative images are shown in Figure 1. For infarct size determination, the collagen deposition in Masson-stained sections was used to define the LV scarred region. The percentage of affected LV wall was calculated through two different validated methods: the area measurement and the midline length measurement by using MIQuant software (Table 6). We found less pronounced fibrosis in Xinmailong and sodium creatine phosphate group than in control group, suggesting Xinmailong and sodium creatine phosphate could protect myocardial tissue from MI induced damage and prevent cardiac fibrosis.

**Figure 1:** Left ventricular myocardial fibrosis (Masson staining 2 × 10 times). **(A)** Sham operation group; **(B)** control group; **(C)** sodium creatine phosphate group; and **(D)** Xinmailong group.

RETRACTED

**Table 6:** Infarction area of Masson staining sections in Figure 1.

Image	Normal area	Infarcted area	LV Lumen area	Infarct size area (%)	Midline length of infarcted region	LV midline length	Infarct size midline length (%)
A	63,533	1,115	15,921	2.29	0	687.71	0
B	40,697	7,973	19,752	16.389	124.42	752.83	16.52
C	31,948	6,186	13,915	16.229	73.31	643.73	11.39
D	41,566	5,462	4,347	11.619	0	542.34	0

To investigate the myocardial protective effect of Xinmailong in detail, we observed the tissue and cellular morphology of left ventricular myocardial cells. Under a light microscope, the myocardial cells in the sham operation group were normal, and no myocardial necrosis was observed. The myocardial infarction in the control group was extensive, and the myocardial necrosis was obvious. Necrosis caused by myocardial infarction in the sodium creatine phosphate group was localized, and normal myocardial cells can be seen around the infarct area. The boundary between the infarct and the surrounding normal myocardial tissue was not clear. A small amount of normal myocardial tissue could be observed in the middle of the necrotic myocardial tissue. Similar with creatine phosphate group, the myocardial infarction was limited in the Xinmailong group. Some normal myocardial tissue existed in the necrotic myocardial tissue, and the myocardial cells surrounding the infarct were normal. The boundary between the infarct and the surrounding tissue was blurred (Figure 2).

**Figure 2:** Left ventricular myocardial infarct size (HE staining 2 × 10 times). **(A)** Sham operation group; **(B)** control group; **(C)** sodium creatine phosphate group; and **(D)** Xinmailong group. Arrows in **(B–D)** indicate myocardial necrosis.

We observed the myocardial tissue arrangement on 20 × 10 magnified HE staining samples. In the control group, the myocardial cells were apparently disordered, and the tissue structure was loose. In the sodium creatine phosphate group, some cardiomyocytes were necrotic, and the myocardial cells in the necrotic site were disorderly arranged. Nonetheless, some normally arranged cardiomyocytes could be observed. The necrotic site had a loose tissue structure. In the Xinmailong group, some normal cardiomyocytes were visible around the necrotic tissue, and the tissue structure was relatively complete (Figure 3).

**Figure 3:** Left ventricular myocardial cell arrangement (HE staining 20 × 10 times). **(A)** Sham operation group; **(B)** control group; **(C)** sodium creatine phosphate group; and **(D)** Xinmailong group.

We then observed the myocardial cell structure more closely. As shown in Figure 4, in the sham operation group, the myocardial cells were intact, and the morphology of the cell membrane, nucleus, and the myofilament arrangement were normal. Myocardial cell necrosis, abnormal nuclear morphology, visible tissue fragmentation, disordered cell arrangement, and loose tissue structure were appeared in the control group. In the sodium creatine phosphate group, the cell arrangement was disordered, the nuclear morphology was abnormal, the tissue structure was loose, and necrotic myocardial cells were visible, but the myocardial cells were partially necrotic and fragmented. In the Xinmailong group, nuclear deformation of necrotic myocardial cells and cell fragmentation were also found, but partially necrotic myocardial cells and some normal cardiomyocytes could be observed around the necrotic cardiomyocytes.

RETRACTED

**Figure 4:** Left ventricular myocardial cell structure (HE staining 40 × 10 times). **(A)** Sham operation group; **(B)** control group; **(C)** sodium creatine phosphate group; and **(D)** Xinmailong group.

To understand the possible mechanism of the Xinmailong’s protective effect. The ultrastructure of myocardial cells was observed using a transmission electron microscope. As shown in Figure 5, in the sham operation group, the myocardium was arranged neatly, the myofibrils were arranged in parallel, the myocyte membrane was intact, the mitochondrial membrane was intact, and the cristae was parallel. In the control group, the myocardial fibers were not arranged neatly, and some collagen and mitochondrial fragments could be visible, suggesting myocardial cell destruction. Apparent abnormalities such as myofilament misarranged and myocardial mitochondrial swelling were also observed in the sodium creatine phosphate and Xinmailong groups, however, the severity was significantly lower than that in the control group. The difference between the phosphocreatine and Xinmailong groups was not significant (Figure 5).

**Figure 5:** Myocardial ultramicroscopic results (2 μm). **(A)** Sham operation group; **(B)** control group; **(C)** sodium creatine phosphate group; and **(D)** Xinmailong group. Arrows in **(B–D)** indicate collagen and mitochondria fragments.

Taken together, these data suggest that both sodium creatine phosphate and Xinmailong apparently protect myocardial cell and accelerate myocardial tissue repair.

## Discussion

The incidence, prognosis, and outcomes of AMI have been greatly improved with the development of society, medical science, and technology (Wang et al., 2017). However, AMI has become a major problem in social development and population health in China. It has the characteristics of acute onset, rapid development, and poor prognosis, seriously threatening human health (Roth et al., 2017). Therefore, urgent attention should be paid to the prevention and treatment of AMI.

RETRACTED

Previous studies showed that patients with AMI had higher levels of inflammation, and the inflammatory response further aggravates myocardial damage (Oliveira et al., 2018). The myocardial tissue damage reduces cardiac function and induces ventricular remodeling (Lin et al., 2018). Xinmailong injection is a compound containing peptides, nucleosides, and complex amino acids extracted from American cockroaches. It has strong diuretic and anti-ischemic effects, improves neuroendocrine imbalance, and protects against HF. In this study, the classic left anterior descending coronary artery ligation was adopted to establish the AMI model in rats. This animal model has the advantages of good stability, high modeling success rate, and high reproducibility. Blood routine and coagulation index was measured after treatment, and no statistically significant difference was found in the liver and kidney function indexes between the Xinmailong group and the control group, suggesting that Xinmailong injection is largely safe.

The thromboelastography showed that the K value was significantly decreased and the angle value was significantly increased in all myocardial infarction groups, including the control, sodium creatine phosphate, and Xinmailong group, compared with the sham operation group, which might be related to the anterior descending branch ischemia. Post-local thrombosis might also be involved and needs to be clarified in future studies.

The inflammatory response is one of major causes of myocardial damage. The levels of inflammatory factors and chemokines in the myocardial tissue are elevated rapidly after myocardial injury in AMI, further exacerbate the inflammatory response and aggravate myocardial infarction, ventricular remodeling, and other forms of cardiac dysfunction (Ahmed et al., 2018). In this study, the levels of inflammatory factors CRP, and myocardial markers such as CK and CK-MB, were significantly lower in the Xinmailong group compared with the control group, suggesting that Xinmailong injection has certain anti-inflammatory effects and protect against myocardial damage. The anti-myocardial ischemia effect of Xinmailong may be related to the antiplatelet aggregation. Some research showed that platelet adherence to immobilized collagen-coated surfaces was decreased by Xinmailong and it inhibited collagen-, thrombin-, and AA-induced platelet aggregations in a dose-dependent fashion (Wang et al., 2019). In addition, Xinmailong was reported to reduce myocardial expression of hypoxia-induced factor-1α (HIF-1α) and decrease plasma endothelin-1 (ET-1) levels, so as to alleviate hypoxia-ischemic myocardial injury (Qi et al., 2017).

RETRACTED

Hemodynamics is a comprehensive manifestation of many factors, such as cardiac systolic function, valve activity, venous return, and ventricular ejection. It is also a specific manifestation of myocardial ischemia. Long-term myocardial ischemia leads to weakened and lost contraction of necrotic areas, and myocardial contraction abnormalities occur (Lefieux et al., 2016). LVSP and +dP/dtmax are sensitive indicators reflecting cardiac systolic function. They are sensitively influenced by myocardial contractility and are important indicators for evaluating myocardial contractility. −dp/dtmax refers to the maximum velocity of isovolumic diastolic left ventricular pressure, which is mainly reflecting the diastolic function of the left ventricle. This study showed that the cardiac function levels decreased to some extent in the other groups compared with the sham operation group, which was related to the modeling of myocardial infarction. However, the hemodynamic parameters were significantly improved in the Xinmailong and sodium creatine phosphate groups compared with the control group, suggesting that both drugs improved the heart function of rats with cardiac insufficiency after myocardial infarction. The LVSP was higher in the Xinmailong group compared with the sodium creatine phosphate group, suggesting that Xinmailong increase myocardial contractility and enhance cardiac function, and its effect was similar to or was even slightly better than that of sodium creatine phosphate. However, the level of LVSP was related not only to left ventricular systolic function, but also to factors such as peripheral vascular resistance. Further studies are needed to confirm this change. At the same time, the BNP level was significantly lower in the Xinmailong and sodium creatine phosphate groups compared with the control group, which further confirmed that Xinmailong injection was similar to sodium creatine phosphate in improving cardiac function.

The pathomorphological changes in the myocardial tissue are the most intuitive indicators reflecting myocardial ischemic injury (Tseliou et al., 2016). The improvement in myocardial pathology is the most solid evidence for the treatment of ischemic injury. Under light microscope, the sham operation group showed intact cardiomyocytes, normal cell membrane, nuclear morphology, and myofilament. The myocardial cells in the control group were necrotic, the nucleus was abnormal, and tissue fragmentation was observed. The cells were arranged in a disorderly manner, and the tissue structure was loose. In the Xinmailong and sodium creatine phosphate groups, the myocardial cells were partially necrotic. The necrotic cardiomyocytes were nucleated, and some normal cardiomyocytes were observed around the necrotic cardiomyocytes. The fibrotic response is essential for maintaining the structure of the heart and preserving cardiac function in response to injury (Meredith et al., 2015). Under the microscope, significantly increased myocardial collagen were observed in control group rats, which was broken and arranged in a disordered collagen fiber content network around the myocardial cells. In Xinmailong or sodium creatine phosphate group, the amount of collagen was less than in control group, suggesting that Xinmailong inhibits the accumulation of collagen. Transmission electron microscopy showed that the myocardial filaments were arranged as neatly in the Xinmailong and phosphocreatine groups as in sham group, and mitochondrial swelling was observed in the myocardium. The degree of tissue damage was not different between the Xinmailong and phosphocreatine group, but was significantly reduced compared with the control group. This result suggests that Xinmailong protect the myocardial cell membrane and alleviate myocardial cell damage, and its protective effect is not inferior to that of creatine phosphate. All in all, our preliminary results suggest that Xinmailong has cardioprotective and anti-inflammatory effects, and it reduce myocardial cell damage, enhance myocardial contractility, and improve cardiac function, while being highly safe. However, Xinmailong’s impact on coagulation function requires further investigation.

RETRACTED

## Data Availability Statement

The original contributions presented in the study are included in the article/supplementary material, further inquiries can be directed to the corresponding author.

## Ethics Statement

The animal study was reviewed and approved by Animal Experimental Center of PLA General Hospital.

## Author Contributions

QS and KL were involved in the concept and design. WZ, KL, YD, JR, and HW were involved in the acquisition of data and analyzed the data. WZ, KL, YD, and QS drafted the manuscript and performed the critical revision of the study. All authors contributed to the article and approved the submitted version.

### Conflict of Interest

The authors declare that the research was conducted in the absence of any commercial or financial relationships that could be construed as a potential conflict of interest.

## References

[ref1] AhmedS. F.ShabayekM. I.Abdel GhanyM. E.El-HefnawyM. H.El-MesallamyH. O. (2018). Role of CTRP3, CTRP9 and MCP-1 for the evaluation of T2DM associated coronary artery disease in Egyptian postmenopausal females. PLoS One 13:e0208038. 10.1371/journal.pone.0208038, PMID: 30557342PMC6296499

RETRACTED

[ref2] FoxK. A. (2000). Coronary disease. Acute coronary syndromes: presentation—clinical spectrum and management. Heart 84, 93–100. 10.1136/heart.84.1.93, PMID: 10862599PMC1729422

[ref3] HanX. N.QiaoS. B.GeJ. B.HanY. L.ChenJ. Y.YuanZ. Y.. (2020). Long-term follow-up of antithrombotic management patterns in patients with acute coronary syndrome in China. J. Geriatr. Cardiol. 17, 246–255. 10.11909/j.issn.1671-5411.2020.05.008, PMID: 32547607PMC7276310

[ref4] LefieuxA.AuricchioF.ContiM.MorgantiS.RealiA.TrimarchiS. (2016). “Computational study of aortic hemodynamics: from simplified to patient-specific geometries” in Advances in computational fluid-structure interaction and flow simulation. eds. BazilevsY.TakizawaK. (Springer International Publishing), 397–407.

[ref5] LinY.WangQ.SongS.ShenJ.WangX. (2018). Effect of humidified oxygen therapy with xiexiang formula on myocardial injury markers and pathological morphology of cardiopulmonary tissue of mice with myocardial infarction. J. Nanjing Univ. Tradit. Chin. Med. 34, 185–189. 10.14148/j.issn.1672-0482.2018.0185

[ref6] LiuS.LiY.ZengX.WangH.YinP.WangL.. (2019). Burden of cardiovascular diseases in China, 1990–2016: findings from the 2016 global burden of disease study. JAMA Cardiol. 4, 342–352. 10.1001/jamacardio.2019.0295, PMID: 30865215PMC6484795

[ref7] LuX.ZhangL.WangJ.LiuH.LiH.ZhouH.. (2018). Clinical efficacy and safety of Xinmailong injection for the treatment of chronic heart failure: a meta-analysis. Front. Pharmacol. 9:810. 10.3389/fphar.2018.00810, PMID: 30140225PMC6094981

[ref8] MeredithA.BoroomandS.CarthyJ.LuoZ.McManusB. (2015). 1,25 Dihydroxyvitamin D3 inhibits TGFbeta1-mediated primary human cardiac myofibroblast activation. PLoS One 10:e0128655. 10.1371/journal.pone.0128655, PMID: 26061181PMC4462580

[ref9] OliveiraJ. B.SoaresA.SpositoA. C. (2018). Inflammatory response during myocardial infarction. Adv. Clin. Chem. 84, 39–79. 10.1016/bs.acc.2017.12.002, PMID: 29478516

[ref10] QiJ.YuJ.TanY.ChenR.XuW.ChenY.. (2017). Mechanisms of Chinese medicine Xinmailong’s protection against heart failure in pressure-overloaded mice and cultured cardiomyocytes. Sci. Rep. 7:42843. 10.1038/srep42843, PMID: 28205629PMC5311956

[ref11] ReynoldsK.GoA. S.LeongT. K.BoudreauD. M.Cassidy-BushrowA. E.FortmannS. P.. (2017). Trends in incidence of hospitalized acute myocardial infarction in the cardiovascular research network (CVRN). Am. J. Med. 130, 317–327. 10.1016/j.amjmed.2016.09.014, PMID: 27751900PMC5318252

[ref12] RothG. A.JohnsonC.AbajobirA.Abd-AllahF.AberaS. F.AbyuG.. (2017). Global, regional, and national burden of cardiovascular diseases for 10 causes, 1990 to 2015. J. Am. Coll. Cardiol. 70, 1–25. 10.1016/j.jacc.2017.04.052, PMID: 28527533PMC5491406

RETRACTED

[ref13] TangX. (2008). Cardiovascular action and therapeutic effect of Xinmailong injection for treating heart failure. Chinese J. New Drug 17, 461–464.

[ref14] TseliouE.KanazawaH.DawkinsJ.GalletR.KrekeM.SmithR.. (2016). Widespread myocardial delivery of heart-derived stem cells by nonocclusive triple-vessel intracoronary infusion in porcine ischemic cardiomyopathy: superior attenuation of adverse remodeling documented by magnetic resonance imaging and histology. PLoS One 11:e0144523. 10.1371/journal.pone.0144523, PMID: 26784932PMC4718597

[ref16] WangX. Y.HuangX. M.YangW. D.ZhengP. (2017). Effects of antioxi-dant therapy on prevention and trearment of ventricular re-modeling in patients with acute myocardial infarction. Chin. Hosp. Pharm. J. 37, 1182–1184. 10.13286/j.cnki.chinhosppharmacyj.2017.12.15

[ref15] WangH.YeY.WanW.WangL.LiR.LiL.. (2019). Xinmailong modulates platelet function and inhibits thrombus formation via the platelet alphaIIbbeta3-mediated signaling pathway. Front. Pharmacol. 10:923. 10.3389/fphar.2019.00923, PMID: 31507419PMC6716460

